# Value of Rehabilitation Training for Children with Cerebral Palsy Diagnosed and Analyzed by Computed Tomography Imaging Information Features under Deep Learning

**DOI:** 10.1155/2021/6472440

**Published:** 2021-07-20

**Authors:** Xi Zhang, Zhenfang Wang, Jun Liu, Lulin Bi, Weilan Yan, Yueyue Yan

**Affiliations:** ^1^Department of Rehabilitation, Children's Hospital of Shanxi Province, Taiyuan 030025, Shanxi, China; ^2^Outpatient Department of Infectious Diseases, Children's Hospital of Shanxi Province, Taiyuan 030025, Shanxi, China; ^3^Imaging Department of CT Room, Children's Hospital of Shanxi Province, Taiyuan 030025, Shanxi, China

## Abstract

To analyze the brain CT imaging data of children with cerebral palsy (CP), deep learning-based electronic computed tomography (CT) imaging information characteristics were used, thereby providing help for the rehabilitation analysis of children with CP and comorbid epilepsy. The brain CT imaging data of 73 children with CP were collected, who were outpatients or inpatients in our hospital. The images were randomly divided into two groups. One group was the artificial intelligence image group, and hybrid segmentation network (HSN) model was employed to analyze brain images to help the treatment. The other group was the control group, and original images were used to help diagnosis and treatment. The deep learning-based HSN was used to segment the CT image of the head of patients and was compared with other CNN methods. It was found that HSN had the highest Dice score (DSC) among all models. After treatment, six cases in the artificial intelligence image group returned to normal (20.7%), and the artificial intelligence image group was significantly higher than the control group (*X*^2^ = 335191, *P* < 0.001). The cerebral hemodynamic changes were obviously different in the two groups of children before and after treatment. The VP of the cerebral artery in the child was (139.68 ± 15.66) cm/s after treatment, which was significantly faster than (131.84 ± 15.93) cm/s before treatment, *P* < 0.05. To sum up, the deep learning model can effectively segment the CP area, which can measure and assist the diagnosis of future clinical cases of children with CP. It can also improve medical efficiency and accurately identify the patient's focus area, which had great application potential in helping to identify the rehabilitation training results of children with CP.

## 1. Introduction

Cerebral palsy (CP) is one of the common causes of disability in children. It is the brain tissue damage caused by the immature brain (fetal period to within one year of life) due to congenital malformations or hypoxia, trauma, infection, and other factors after birth, which further causes a group of neurological syndromes in children with nonprogressive movement abnormalities and postural abnormalities as the main manifestations, accompanied by cognition, sensory, and communication disorders and other complications [1]. With the continuous development of perinatal medicine and neonatal life support technology and the improvement of rescue technology, more and more ultrapremature babies are able to survive. These premature babies are extremely immature and face severe challenge such as breathing, nutrition, metabolism, and infection. Their brain damage easily occurs, CP is caused, and the risk of disability is increased [2, 3]. Neuroimaging examination is an important auxiliary examination for central nervous system damage, which can provide objective basis for changes in tissue morphology for clinical diagnosis and treatment. The traditional cranial CT has been widely used in the cranial imaging examination of children with CP and has accumulated certain experience [4]. The other functional imaging examinations developed based on traditional techniques such as magnetic resonance imaging (MRI), ultrasound (US), positron emission tomography (PET), and other devices can assess the function of brain tissue through local blood flow changes, water molecular activity, and metabolic status. The lesions associated with the occurrence of CP were mapped in more detail to provide evidence of functional and metabolic abnormalities for some lesions with insignificant morphological changes. Up to now, medical imaging is an indispensable part of the clinic, and it plays an irreplaceable role in diagnosis and treatment. However, the workload of doctors is huge. Studies showed that, in some cases, general radiologists must make a diagnosis every three to four seconds in an 8-hour working day to meet the needs of the workload [5]. The accuracy of doctors' diagnosis results will be greatly affected by such a large work intensity, and misdiagnosis and missed diagnosis will be caused. However, there are also obvious problems in the current study. (I) The commonly used brain images have millimeter resolution. However, some diseases do not cause significant structural changes and require high resolution and small-scale brain imaging techniques. (II) The sample data only contains a certain kind of special diseases and health data. In actual diagnosis, the patient may suffer from ten related diseases. (III) The excessive number of extracted features consumes a large amount of storage space and at the same time greatly increases the computational complexity and leads to dimensional disaster. (IV) The classification accuracy should be further improved to meet the requirements of practical use. (V) The generalization performance of the classifier is poor, and the prediction effect of the new samples is obviously lower than that of the training samples.

With the development of artificial intelligence (AI), people began to try to use computer technology to assist doctors in diagnosis, which produced a computer-aided diagnosis (CAD) [6]. Taking the most widely used mammography CAD screening as an example, more than 74% of mammograms in the United States were performed with the aid of the CAD system by 2010 [7]. However, the advantages of CAD were questionable; several large trials concluded that there was little benefit from CAD. The accuracy of radiologists' diagnoses was reduced; thus high biopsy rates were caused. To eliminate the false alarms generated by these systems, the diagnostic process becomes more complex [8]. At present, diagnosis based on medical imaging mainly relies on radiologists' manual review of images and manual analysis of radiological images. This is a very time-consuming work, requiring radiologists to consult hundreds of sections and multiple lesions through three-dimensional CT scanning equipment [9]. For early detection, detecting lesions that are “too small to characterize” is particularly important, which requires time and effort on the part of the radiologist. In addition, the increasing huge amount of image data also brings great challenges for image reading. To effectively improve the efficiency of medical image reading, reduce the error rate of diagnosis, and provide effective auxiliary information for imaging physicians, the auxiliary diagnostic technology based on intelligent image analysis is becoming more and more important. In recent years, computer-aided diagnosis based on intelligent image analysis has gradually become a research hotspot in the medical field. Artificial intelligence algorithms have been used in the field of medical image data analysis and processing. By integrating these algorithms into clinical practice, effective and accurate diagnostic results are obtained. The traditional method of intelligent imaging diagnosis compares the automatically labeled or segmented area with the predefined benchmark template, but it still needs the imaging expert to give the final diagnosis result. In the application of disease diagnosis, abdominal CT imaging is the most important imaging means in the clinical diagnosis and follow-up of tumor diseases, which is widely used in the detection, segmentation, and diagnosis of lesions. Since different types of lesions correspond to different characteristics, how to separate the lesion area from the image is the key to the success of the high-precision diagnosis system [10]. To improve the accuracy of the automatic diagnosis system, the medical image assisted diagnosis system based on artificial intelligence mainly includes four aspects as follows: (I) image preprocessing, which improves the image quality and enhances the contrast of lesions; (II) detection and segmentation of the region of interest (ROI), which reduces the influence of interference background on the system; (III) feature extraction, selection, and classification, which improve the characterization ability of the target; (IV) the semantic segmentation of tumor, which can obtain the semantic features of lesions and improve the accuracy of recognition. The extraction of efficient features in the four key steps of the auxiliary diagnosis system is the core technology of the system. At present, the performance of medical image aided diagnosis system based on shallow learning completely depends on the characterization ability of features and the generalization performance of classification diagnosis model.

In short, the development of AI technology has provided new ideas to solve such medical problems. In particular, multidisciplinary knowledge such as radiology and computer science was integrated by imaging omics. High-throughput features can be mined from medical images and modeled and analyzed to provide clinical decision support for rehabilitation training for children with CP.

## 2. Methods

### 2.1. Research Object

Children with CP who were outpatient or hospitalized in our hospital from June 2017 to June 2020 were taken as research subjects. A total of 73 cases met the requirements; 44 were males and 29 were females. The age range was 1 to 14 years and the average age was 47.7 ± 37.2 months.

The classification was carried out according to the gross motor function classification system (GMFCS) [11]. There were 8 cases of GMFCS I (4 males, 4 females), 21 cases of GMFCS II (12 males, 9 females), 23 cases of GMFCS III (13 males, 10 females), 11 cases of GMFCS IV (8 males, 3 females), and 10 cases of GMFCS V (7 males, 3 females).

#### 2.1.1. Inclusion Criteria

The abovementioned children met the diagnostic criteria for CP and must meet the following four necessary conditions: (a) nonprogressive aggravating dysfunction that persisted, which was caused by central nervous system damage; children with complications such as muscle damage and joint deformation as the course of CP was prolonged; (b) children with deviations in motor development and abnormal postures (motor development was included or not included); (c) the original reflex not disappearing or the erection reflex and balance response delayed or absent, which may be accompanied by a positive pathological reflex; (d) children with abnormal muscle tone and strength. In addition, there were two reference conditions whether it met the diagnosis of CP: (a) children with a history or risk factors that cause CP; (b) children with cranial imaging evidence.

#### 2.1.2. Exclusion Criteria

The exclusion criteria included (a) the diagnosis of abnormal motor development in children that was consistent with general developmental retardation and developmental coordination disorder; (b) children with induced epileptic seizures caused by acute ketoacidosis, water and electrolyte disorders, acute brain injury, febrile convulsions, hypoglycemia, and drug poisoning, etc.; (c) children with metal implants or other contraindications for CT examination; (d) children with abnormal motor function caused by other genetic metabolic reasons; (e) children with motor dysfunction and epileptic seizures caused by tumors, peripheral neuropathy, and genetic metabolic diseases, etc.

A total of 73 children with CP met the above inclusion criteria and were included in the research. The research had been approved by the medical ethics committee of *X* hospital, and the informed consent form had been signed by the families of the children involved in the research.

### 2.2. Experimental Equipment

74 contrast-enhanced CT samples constituted the dataset of the research. The Philips Brilliance 1281 CT scanner (Philips Healthcare, Amsterdam, Netherlands) was used. The tube voltage and current were 120 kV and 220 mA, respectively, the size of the collimator was 64 × 0.625 mm, and the Fov was 20 × 20 cm. The 512 × 512 size imaging matrix was used, the pixel size range was 0.58 to 0.98 mm, and the reconstruction interval was 5 mm. All scans were manually segmented by two radiologists using Itk snap software (version 3.4; http://www.itksnap.org), and the segmentation differences were resolved through discussion until a consensus was reached. The data set was randomly divided into three subsets, and 84, 20, and 30 samples were included for training, verification, and testing, respectively.

### 2.3. Experimental Environment

#### 2.3.1. CNN Model

The proposed CNN model is shown in Figure 1, which was similar to 3D U-NET. The image features can be extracted layer by layer by the encoder, and the segmentation map can be generated by the decoder. The 3D U-Net was modified to be suitable for this task. In the original 3D U-Net, there were two 3 × 3 × 3 convolutions included in each level, which was replaced by two modules. To reduce the size of the feature map, the step S3D convolution was used to replace the pooling operation. The goal of the decoder was generating high resolution feature maps. First, the feature graph was upsampled, and then the upsampled feature graph was cascaded with the feature graph from the corresponding level of the encoder. After cascading, the MSC module was used to adjust the number of feature graphs. The lightweight 3D CNN had fewer parameters and computational costs compared to the original 3D U-NET.

#### 2.3.2. Deep Learning Mode

The Python deep learning framework was used to write code, which was trained on NVIDIA GeForce GTX 1080TIGPU. There were 100 training cycles and the training time was about 12 hours. The Adam optimizer was used with an initial learning rate of 0.001. The GDL loss function similar to the previous chapter was used to optimize network parameters. If the validation set loss was not decreased in the last 20 training cycles, the learning rate was reduced to 1/5 of the original. The rotation, scaling, deformation, mirroring, and other data were not used to enhance technology to focus on the impact of network structure. The LeakyReLU was used as the activation function. The negative part of the feature information can be retained by LeakyReLU to prevent falling into a local minimum compared with the standard ReLU. For 2D CNN, batch normalization was used to reduce internal covariant offset problems. For 3D CNN, a number of criteria were calculated using instance normalization as performance indicators to quantify the segmentation results, including DSC, sensitivity, and positive predictive value (PPV).

### 2.4. Comparative Test with 3DCNN Method

Compared with the 3D CNN method, each CT was first resampled to 256 × 256 × 64 to maximize the utilization of 11 GB of GPU memory. In the decoder, each layer was composed of a trilinear upsampling layer with a factor of two, followed by two 3 × 3 × 3 convolutions, and instance normalization and LeakyReLU were used to activate each layer. The jump connection was used to provide the decoder with spatial information from the encoder. Finally, the nearest neighbor sampling was used to upsample the segmentation result to the size of 512 × 512 × 64.

### 2.5. Treatment Methods

The physical therapy (PT), occupational therapy (OT), and speech therapy (ST) were used as the main treatment methods. The selected method was Bobath's method to suppress the abnormal posture, abnormal posture reflex, and abnormal movement patterns of children with CP. The facilitating techniques were used to promote cervical erection, sitting erection, standing erection, and static and dynamic balance in children with CP. The German Voyt method was selected to perform reflex movement of the body to promote normal motor development and induce training with reflex turning over and reflex abdominal crawling. According to the child's condition, one-to-one rehabilitation training was carried out by the rehabilitation therapist. The training was one to two hours a day, and 90 days was a course of treatment. The rehabilitation training for children with mild CP was one to two courses, and the rehabilitation training for children with severe CP was three to four courses.

### 2.6. Observation Indicators

Before and after treatment, the cerebral artery blood flow velocity (VP) and the vascular pulse index (PI) of the children in both groups were examined by Libong CBC-II transcranial doppler (TCD) cerebrovascular ultrasound to understand the recovery of cerebral blood circulation. The routine EEG and single photon emission cranial computed tomography (SPELT) were performed before and after treatment to assess cerebral perfusion and neuronal functional status. The CT scans of the head were performed after three to six months of treatment to observe the morphological and structural recovery of the brain. The development quotient (DQ) of the children was assessed using the Geisel method to assess the children's social adaptability, personal social ability, language ability, general motor, and fine motor recovery before and after treatment.

### 2.7. Statistical Analysis

SPSS 20.0 was used for statistical analysis of the data. Measurement data such as body weight and scores were expressed as mean ± standard deviation, and *t*-test was used to compare the data of normal distribution between the two groups. When three groups or more were compared, analysis of variance was carried out first, and then pairwise comparison was made. Enumeration data were expressed as percentage (%), and comparison between two groups was performed by *χ*^2^ test or corrected *χ*^2^ test. *P* < 0.05 was considered statistically significant.

## 3. Results

### 3.1. Comparative Test with 2DCNN Method

It was compared with 2D CNN method. The 2D models allowed larger images as input than 3D models (Figure 2). Therefore, full-resolution CT slices were used to collect detailed contextual information. The 2D CNN similar to 3D CNN was constructed, and the difference was that 3D convolution was replaced with 2D convolution. The 3D trilinear upsampling layer was replaced with 2D bilinear upsampling layer, and batch normalization was used in convolution.

### 3.2. Segmentation Results in Different Ways

Figures 3 and 4 show the segmentation results of 2D CNN and 3DCNN on the test set, respectively. The blue represented the gold standard for segmentation, and the red represented the result of automatic segmentation. These segmentation results indicated that 3D CNN can segment cancer regions more accurately than 2DCNN.

### 3.3. Comparative Experiment of Loss Correspondence Teaching

The choice of loss function was crucial to obtain accurate segmentation results when dealing with serious category imbalance. The GDL loss function was used to solve the class imbalance problem in CT images. Since many works proved that Dice loss can obtain more reliable results than cross-direction loss, there was a performance difference between Dice loss and GDL loss. Figures 5 and 6 show the average DSC on the validation set, and the loss of the model trained with GDL was smaller than the loss of the model trained with Dice. The DSC curve of the model's validation set was smoother when GDL was used for training, which indicated that GDL was more stable for CT image segmentation.

### 3.4. Quantitative Results of the Test Set

Figure 7 shows the quantitative results of the test set. The model with Dice loss training had lower DSC, lower PPV, and higher sensitivity compared with HSN, but all the deviations were large. The results showed that the problem of category imbalance can be effectively solved by GDL.

### 3.5. Spatial Convolution Contrast Experiment

The goal of 2D CNN was providing fine-grained semantic information about smaller and less salient objects for accurate segmentation. Therefore, the high spatial resolution must be retained in the output feature map. A simple reduction of the pooled or stepped convolution layer resulted in a reduction of the receptive field. Therefore, the cavity convolution was proposed to enlarge the receptive field and the resolution of the feature map was maintained. To study whether the hole convolution helped to learn fine-grained semantic information, it was compared with the standard 2D convolution version (HSN-N). The standard 2D convolution version (HSN-N) had the same architecture as HSN, but all 2D convolution layers did not use hole convolution. The convolution kernels with large void ratios may be too sparse to capture local features, which led to the “grid problem.” To investigate the effect of large void rate on segmentation performance, another HSN model (2D HSN-L) with larger void rate was evaluated. The void rate of the original HSN was increased from three to five by this model.  Figure 8 shows the qualitative segmentation results of different experiments on the test set. The blue represented the gold standard, and red represented the result of automatic segmentation. These segmentation results showed that HSN performed well in segmenting lung cancer even in a small area. This was because the model can learn remote 3D context information and fine-grained 2D semantic information.

### 3.6. Results of Children's Rehabilitation Data

The SPECT examination showed hypoperfusion of cerebral blood flow and decreased functional activity of neurons in the treatment group before treatment, and 27 cases returned to normal after treatment (96.4%). There were 29 cases of hypoperfusion of cerebral blood flow and decreased functional activity of neurons in the control group before treatment, and 6 cases returned to normal after treatment (20.7%). The return to normal rate of SPECT in the treatment group was significantly higher than that in the control group (XPINGFANG = 33 5191, *P* < 0.001). The cerebral hemodynamic changes of the two groups of children before and after treatment showed that VP of the cerebral artery in children was (139.68 ± 15.66) cm/s after treatment, which was significantly faster than that before treatment (131.84 ± 15.93) cm/s, *P* < 0.05. The cerebral artery PI of the children was 0.91 ± 0.19 after treatment, which was significantly lower than that of 1.18 ± 0.24 before treatment, *P* < 0.05. However, in the control group, the cerebral artery VP and PI of the children had no significant difference before and after treatment, *P* > 0.5. After treatment, there were significant differences in VP and PI between groups (*P* < 0.05). The changes in DQ of the two groups of children before and after treatment are shown in Figure 9. The difference of GM FM scale scores before and after treatment in the two groups of children is shown in Figure 10.

## 4. Discussion

A large amount of image data was generated in the process of diagnosis and treatment of CP lesions. These data were usually subjectively evaluated by doctors based on experience, and then the corresponding diagnosis and treatment plan were made. However, the features observed by doctors with only naked eyes from image data were very limited, and the potential of image data was often not fully utilized. For many years, the quantitative information that was not available to the human eye was extracted by many scholars with the help of complex mathematical and statistical algorithms, based on which the corresponding diagnosis and treatment plan were carried out, and even the progress of the disease was predicted. The image omics came into being with the development of AI technology. The machine learning algorithms were used to mine high-throughput features from medical images and perform modeling analysis [12]. More and more evidence showed that imaging omics can be used for the quantitative characterization of CP lesions for the diagnosis, treatment planning, and prognosis of the disease. Thus, an important research direction of AI technology in the field of medical applications was constituted [13–17].

In recent years, with the rise of deep learning technology and computer vision technology, it has become more and more urgent to develop automatic segmentation algorithms with high accuracy and high stability [9]. The problem of CT image segmentation was studied based on the brain MRI and lung CT images and the use of deep learning technology. In addition, for the grading of brain lesions, the impact of deep learning segmentation results and manual segmentation results on imaging omics research was compared in the research. For the prediction of chemotherapy outcomes in patients with CP, imaging omics models were also constructed and analyzed in combination with clinical features. The reproducibility of imaging omics research was still an unresolved problem, and the clinical application of imaging omics was greatly affected by this problem. Studies showed that more than 90% of research had not undergone rigorous external verification and lacked multicenter diversity data [18, 19]. A hybrid segmentation network based on deep learning (HSN) was used for CT brain image segmentation and the accuracy of image analysis of brain cell function in children with CP can be improved. The language function, motor function, cognitive function, language quotient, great motor development quotient, fine motor development quotient, personal social, and social adaptation development of the brain of children with CP in the HSN group were significantly improved after treatment compared to before treatment.

In this research, a hybrid segmentation network HSN based on deep learning was proposed for CT brain tissue image segmentation. CT images often have higher resolution than MRI images. How to segment CT images effectively is always a difficult problem. HSN can effectively solve this problem. HSN includes a lightweight 3D CNN and a refined 2D CNN. 3D CNN uses desampled images and spatiotemporal separable 3D convolution to reduce memory requirements and computational costs. 2D CNN can learn fine-grained semantic information while maintaining a high spatial resolution. A hybrid feature fusion module was proposed to effectively integrate 2D and 3D features. This network structure combines the advantages of 3D CNN learning long-range contextual information and 2D CNN learning semantic information. The results showed that this model can segment CP lesion area accurately on CT images. The development of deep learning and imaging omics has promoted the progress of medical imaging. Radiology using artificial intelligence can automate certain clinical tasks to some extent. In addition, it can reduce the heavy workload of doctors and improve the diagnostic efficiency, so as to optimize the allocation of social medical resources. However, there are still some shortcomings, which need to be further strengthened in the future. For example, traditional image omics feature extraction methods have certain limitations without adoption of deep learning in feature extraction. Deep learning methods, especially CNNs, can learn rich texture information from medical images in a hierarchical manner. Deep features have a more powerful feature representation than hand-designed features. In the future work, we will carry out related studies on feature extraction based on deep learning to further explore the potential of image data.

## 5. Conclusion

In this study, a hybrid segmentation network HSN based on deep learning was proposed for CT brain tissue image segmentation. After treatment, six patients in the artificial intelligence group returned to normal (20.7%), which was significantly higher than the control group (*X*^2^ = 335191, *P* < 0.001). Cerebral hemodynamic changes were obvious in both groups before and after treatment. VP of the cerebral artery was (139.68 ± 15.66) cm/s after treatment, which was greatly faster than that before treatment (131.84 ± 15.93) cm/s, *P* < 0.05. In general, the deep learning model can effectively segment the CP area and assist in the clinical case measurement and diagnosis of future CP children. In addition, the deep learning model can improve medical efficiency and accurately identify patients' focal areas, which has great application potential in helping to identify the rehabilitation training results of children with CP.

## Figures and Tables

**Figure 1:** CNN model.

**Figure 2:** The average validation set DSC of 2D CNN and 3D CNN in 100 training cycles.

**Figure 3:** 2D CNN.

**Figure 4:** 3D CNN.

**Figure 5:** Training process of different loss function.

**Figure 6:** The average DSC of the verification set of different loss functions.

**Figure 7:** Quantitative results of the test set.

**Figure 8:** Qualitative segmentation results of different experiments on the test set (red was the artificial segmentation area, and blue was the model segmentation area). (a) HSN; (b) HSN-Dice; (c) HSN-S3D.

**Figure 9:** Changes in DQ of the two groups of children before and after treatment (^*∗*^indicated significant difference.).

**Figure 10:** Difference of GM FM scale scores before and after treatment in the two groups of children (^*∗*^indicated significant difference).

## Data Availability

No data were used to support this study.
